The article "Effect of Physical Exercise Intervention Based on Improved Neural Network on College Students' Mental Health" was published in 2022. Journal: Comput Math Methods Med.

# Effect of Physical Exercise Intervention Based on Improved Neural Network on College Students' Mental Health

**DOI:** 10.1155/2022/4884109

**Published:** 2022-06-21

**Authors:** Linlin Cai

**Affiliations:** Nanjing Medical University, Nanjing, 210000 Jiangsu, China

## Abstract

Physical exercise refers to various physical exercises carried out through certain means and methods. Physical exercise can not only achieve the purpose of strengthening the body and health but also make people face challenges in physical and mental sports, and the resulting psychological satisfaction and excitement make exercisers happy physically and mentally. Physical activity has a certain appeal that makes it one of the most effective ways for modern people to alleviate mental illnesses. The human brain's reaction time is linked to its thinking speed and intelligence. Regular physical activity can increase human brain cell reaction time and completely utilize human brain capacity, which is beneficial to the healthy development of human attention, memory, imagination, and thinking ability. Scientific and reasonable physical exercise is also an important means to improve people's intelligence levels. Everyone's physical health level is closely related to their mental health. A healthy mind comes from a healthy body. A large number of scientific studies have confirmed that reasonably arranging the contents and methods of physical exercise according to their own health level and psychological state cannot only enhance the physique of college students but also cultivate their excellent personality. Firstly, this paper summarizes the influence of physical exercise on mental health. The ways of employing physical exercise to improve and improve the mental health of college students are presented in this study. Then, this paper proposes a physical exercise intervention based on an improved neural network (NN), which has an impact on the mental health level of college students, and the effectiveness of this model is verified by simulation experiments.

## 1. Introduction

Nowadays, with the rapid development of the social economy, the stress events faced by college students will also increase in a complex environment. When people encounter stressful events in life, they will have a sense of stress [1]. When people do not know how to face this sense of pressure, they will have all kinds of negative emotions. The National Health Commission released the content on the development of teenagers' mental health, pointing out that with the rapid development of the economy and society, various complex relationships between adults will involve teenagers, and they will also face environmental changes and complex interpersonal communication, which will put pressure on them [2]. The psychological and physiological development of college students in this period is not fully mature. They are more likely to feel pressure and develop psychological and behavioral difficulties, such as irritation and anxiety, when their living environment changes [3]. In recent years, negative emotions have also received extensive attention in the field of psychology. Previous studies have shown that college students' stress events lead to the rise of psychological pressure, and the impact of the increase of psychological pressure on negative emotions is also gradually increasing [4]. The relationship between physical exercise and students' mental health is shown in Figure 1.

The proportion of negative emotions caused by psychological pressure is as high as more than 20%, mainly because college students are prone to negative emotions such as anger, anxiety, and depression in the face of various stress events [5]. Foreign researchers have found that stress can predict negative emotions; at the same time, some studies have found that the pressure perceived by individuals in daily life can positively predict a series of negative emotions such as worry and anger. Therefore, it is necessary to adopt effective regulation methods to regulate and guide college students' psychological pressure and negative emotions, so as to enhance the development of physical and mental health [6]. Physical exercise, as a means of control, has been demonstrated in some studies to be more sensitive to the impact of individual mood in the field of mental health; both short-term exercise and long-term exercise can alleviate the negative emotional state caused by psychological pressure [7]. In an experimental study, the meta-analysis of the impact of stressors on emotion pointed out that when subjects respond to stressors, their negative emotions will also increase. In daily life, college students' psychological stress, negative emotion, and physical exercise are different [8]. By tracking and measuring them, this paper explores the relationship between college students' psychological stress and negative emotion, and the impact of psychological stress on a negative emotion further enriches the relevant research on the relationship between college students' psychological stress and negative emotion and explores the regulatory effect of physical exercise between psychological stress and negative emotion. It serves as a vital foundation for future daily follow-up study in this sector [9].

This paper proposes a physical exercise intervention based on an improved NN, which has an impact on the mental health level of college students. Track and measure the daily psychological pressure, negative emotion, and physical exercise of college students, understand the overall situation of college students in these three aspects, deeply analyze the relationship between psychological pressure and negative emotion and the impact of psychological pressure on a negative emotion, and explore the regulatory effect of physical exercise on their relationship. At the same time, it puts forward reasonable suggestions for improving college students' psychological pressure and negative emotional state and promoting their physical and mental health.

The arrangements of the paper are as follows: Section 2 discusses the related work.  Section 3 defines the design of application model.  Section 4 examines the experiments and results.  Section 5 concludes the article.

## 2. Related Work

### 2.1. Effect of Sports Intervention on Psychological Stress of College Students

Compared with teenagers, college students enjoy higher freedom of activities. They choose their own way of life according to their own principles, schedules, and likes and dislikes. They can control their leisure time and choose their favorite exercise environment and exercise methods [10]. They can arrange the time according to their own schedule, regularly participate in physical exercise, master the skills needed for lifelong physical exercise, and may eventually become a lifelong sports population. Therefore, it is particularly important to increase the frequency of physical exercise during college. However, research shows that the frequency of physical exercise decreases with age [11]. Generally speaking, from children to teenagers, from teenagers to college students, and from college students to adults, the frequency of physical exercise is getting lower and lower. Researchers conducted a survey on the reasons for the formation of exercise habits among college students. The results found that students who participated in a course on jogging and health knowledge may have a more positive attitude towards physical exercise and are more likely to become a person who adheres to jogging as a way of fitness [12]. The mechanism of physical exercise affecting psychological stress is shown in Figure 2.

Regular physical exercise increases the nerve excitation conduction frequency between brain and muscle, promotes the increase of brain nerve excitation, and then inhibits the level of individual psychological pressure [13]. There is an obvious item effect of sports on psychological stress: it may be related to the item group characteristics of sports. According to the event group theory, football and basketball belong to skill-dominated the same field antagonistic projects. The characteristics of this event group are high exercise intensity, which can make the exerciser focus on the limited stimulus sources during the exercise, and then lose the feeling of time. Integrate oneself organically with the environment so that the body and soul are in a balanced state with a strong sense of control and ability [14].

Volleyball, table tennis, and badminton belong to skill-oriented net separated antagonistic events, which are characterized by strong confrontation and sports load. In the process of exercise, exercisers communicate through body language. The sense of joy after victory or the negative mood after failure makes physical activities stimulate the nervous system, which is conducive to the individual getting rid of the paranoid symptoms of depressed thoughts and delusions [15]. Roller skating belongs to endurance events dominated by physical fitness. This group belongs to aerobic exercise. Aerobic exercise has a good therapeutic effect on mild to moderate anxiety and depression. Wushu belongs to the skill-oriented project, which is difficult to express beauty. The characteristics of the project can improve the flexibility and balance of the exerciser's nervous system, effectively enhance the individual's self-control ability, and significantly promote the adjustment of individual psychological states [16]. Individuals can improve their self-awareness and self-awareness in their interpersonal communication and then adjust their adaptive adjustments in the objective environment, which is crucial in improving individual psychological difficulties and development.

### 2.2. Effect of the Exercise Intervention on College Students' Health Belief

Health belief can not only affect the behavior of individuals participating in physical exercise but also effectively improve the level of individual health belief through sports intervention [17]. There is no systematic research and explanation on the mechanism of sports affecting health belief, but it can be explained according to three theories. First, there is social cognitive theory, which maintains that human activities are the outcome of interactions between people, their behavior, and their surroundings. Individuals increasingly realise the function and importance of physical activity in sports and believe that physical activity can successfully avoid their personal risks and diseases, resulting in an increase in individual health belief [18]. Second, the theory of planned behavior holds that attitude has the function of behavior belief, which enables individuals to perceive the advantages and disadvantages of physical exercise behavior when participating in sports, so as to recognize physical exercise behavior and improve the level of individual health belief [19]. Third, the theory of protective motivation holds that the comprehensive perception of efficacy and response cost produces stress evaluation. When the internal reward and external reward system of individual health behavior perceive that physical exercise can reduce the severity and susceptibility of individual diseases, the comprehensive perception of reward and fear will produce benign evaluation, so as to improve the level of individual health belief [20].

College students' perceptions of physical activity are not limited to certain sports, such as aerobics. This study is significant because it demonstrates that previously acquired knowledge about physical activity and health can be carried over from college to adulthood. In other words, if a person takes physical exercise as an important part of his life in college, this lifestyle is more likely to last for the rest of his life [21]. Then, scholars compared the physical exercise of students from four different universities, which have different requirements for physical education. The results show that the subjects from schools with high requirements for physical education have a higher level of physical exercise than other subjects and are better than other subjects in mastering physical exercise knowledge, attitude towards physical education, and exercise habits. At the same time, the research also shows that subjects from schools with high requirements for physical education are relatively more active in physical exercise and tend to show a high desire for exercise [22]. The impact of an exercise intervention on college students' health beliefs is shown in Figure 3.

### 2.3. Research Status of Improved Neural Network

The NN is a system that simulates the results and functions of the human brain NN. Good self-learning, self-organization, fault tolerance, and the ability to simulate nonlinear relations make NNs widely used in the field of science and technology [23]. It has been proved that a simple three-layer feedforward NN using a sigmoid response function can approximate any nonlinear function. The superior performance of NNs largely depends on the learning of weights [24]. The most widely used weight learning method is the BP algorithm, which uses the response propagation of error to adjust the weight. However, the BP algorithm is powerless for systems that cannot determine gradient information [25].

Many academics have begun to examine utilizing the particle swarm optimization algorithm to alter the weight of NN, and the particle swarm optimization method can also optimize the structure of the NN [26], due to its development as a good global convergence approach that is simple to implement. So far, there are two main methods to train NNs with particle swarm optimization algorithms: to train the weights of NNs with particle swarm optimization algorithms [27]. One is to combine the particle swarm optimization algorithm with the BP algorithm, using the powerful global search ability of the particle swarm optimization algorithm and the good local search characteristics of the BP algorithm [28]. When the particle swarm optimization algorithm converges to a certain degree, the BP algorithm is used to continue to search for the global best of particle swarm optimization and finally get the global optimal solution [29].

## 3. Design of Application Model

### 3.1. Basic Particle Swarm Optimization Algorithm

The particle swarm optimization algorithm updates iteratively from the initial random position until it finds the global optimal position, that is, the global optimal solution of the problem. The particle swarm optimization algorithm is a random search optimization algorithm, which has good global convergence for multimodal problems. The updated formula is as follows:

(1) $$\begin{array}{c} v_{i,d}^{k+1}=v_{i,d}^{k}+c_{1}\times r_{1}\times \left(p_{i,d}^{k}-x_{i,d}^{k}\right)+c_{2}\times r_{2}\times \left(p_{g,d}^{k}-x_{i,d}^{k}\right),\\ x_{i,d}^{k+1}=x_{i,d}^{k}+v_{i,d}^{k+1}. \end{array}$$

The speed update of particle swarm optimization is divided into three parts: the first portion is the particle's speed before iteration; the second part is the cognitive part, which is the particle's best location; and the third part is the social part, which is the particle's best position in the particle group.  Figure 4 depicts the basic flow of the particle swarm optimization technique.

Unless the optimal solution of the problem is on the trajectory of particle swarm optimization, the particle swarm will fly down at the current speed and in the same direction until it hits the edge of the search; particle swarm optimization algorithm cannot find the optimal solution, and the optimal solution must be almost impossible on the trajectory of particle swarm optimization. In order to achieve a better balance between local search and global search, inertia weight factor is introduced into the basic particle swarm optimization algorithm. The mathematical expression is as follows:

(2) $$\begin{array}{c} v_{i,d}^{k+1}=w^{*}v_{i,d}^{k}+c_{1}\times r_{1}\times \left(p_{i,d}^{k}-x_{i,\text{d}}^{k}\right)+c_{2}\times r_{2}\times \left(p_{g,d}^{k}-x_{i,d}^{k}\right). \end{array}$$

The inertia weight factor decreases linearly, as shown below.

(3) $$\begin{array}{c} w\left(k\right)=-0.5\left(\frac{k}{\max\text{ number}}\right)+0.9. \end{array}$$

The decreasing inertia weight factor makes the algorithm has better global search ability in the early stage and better convergence in the later stage, but the convergence speed is relatively slow. The increasing inertia weight factor makes the algorithm to converge quickly in the early stage. The inertia weight factor that increases first and then decreases is shown in the figure below.

(4) $$\begin{array}{c} w\left(k\right)=\left\{\begin{array}{cc} 1\times \frac{k}{\max\text{ number }}+0.4, & 0\leq \frac{k}{\max\text{ number }}\leq 0.5,\\ -1\times \frac{k}{\max\text{ number }}+1.4, & 0.5\leq \frac{k}{\max\text{ number }}\leq 1. \end{array}\right. \end{array}$$

In the whole iterative process, the initial *W* is large, and the particles fly rapidly all over the whole search space. After reaching the iterative threshold, the inertia weight will be limited to FW, and the particles maintain a certain speed to find the global optimal value in the neighborhood of the optimal value. The values of uniformly distributed random inertia weight factors vary according to whether the global optimal particle position changes, as shown in the following:

(5) $$\begin{array}{c} \text{If }\Delta g\text{ best}=0,w=\mathrm{rand}\left(r_{1},r_{2}\right);\text{else }w=\mathrm{rand}\left(r_{3},r_{4}\right). \end{array}$$

The change rate of the optimal fitness value is shown in the following formula.

(6) $$\begin{array}{c} k=\frac{f\left(t\right)-f\left(t-10\right)}{f\left(t-10\right)}. \end{array}$$

The convergence of particles can be seen from its change. If the parameter setting is unreasonable, the speed of particles will increase or decrease rapidly. The ideal velocity of a particle swarm is to start relatively large, get smaller and smaller, and finally become 0. The inertia weight formula is as follows.

(7) $$\begin{array}{c} \left\{\begin{array}{cc} w\left(t+1\right)=\max\left\{w\left(t\right)-\sigma \times \mathrm{rand},w_{\min}\right\}, & v_{\text{ave}}\left(t+1\right)>v_{\text{ideal}}\left(t+1\right),\\ w\left(t+1\right)=\min\left\{w\left(t+1\right)+\sigma \times \mathrm{rand},w_{\max}\right\}, & v_{\text{ave}}\left(t+1\right)\leq v_{\text{ideal}}\left(t+1\right). \end{array}\right. \end{array}$$

When the position of the particle swarm does not change in a continuous number of iterations, the *k*-dimension of the optimal particle position is randomly taken and replaced with a random number with a certain probability. The average particle spacing formula is as follows.

(8) $$\begin{array}{c} D\left(t\right)=\left(\frac{1}{M\cdot L}\right)\overset{M}{\underset{i=1}{\sum }}\;\sqrt{\overset{D}{\underset{d=1}{\sum }}\;{\left(x_{id}^{t}-{\bar{p}}_{d}\right)}^{2}}. \end{array}$$

No matter which mutation operation is adopted, the adaptive mutation operator actually uses an evaluation mechanism to randomly change the position of the optimal particle when the algorithm falls premature. In this case, similar to the multiobjective constraint processing method, all constraint functions are treated as an objective function. When there is a dominant relationship, the multiobjective constraint processing method is used for individual comparison.

### 3.2. Particle Swarm Optimization Improved Neural Network

The NN was trained using the particle swarm optimization approach, which included weight training and structural correction. The optimization problem of finding the ideal continuous weight for NNs is essentially a continuous and difficult optimization problem. However, the possibility of a single restricted infeasible solution in the individual optimal solution may not be the most effective method, because, under this idea, the information of some important infeasible solutions cannot be used, such as the infeasible solutions with small objective function values, which may be closer to the global optimal solution than some feasible solutions. Therefore, it is very necessary to allow the infeasible solution as the guiding position with a certain probability under certain conditions. When using the particle swarm optimization algorithm to train the weights of the NN, the first is the coding of particle swarm optimization, as shown in Figure 5.

The position of each particle represents the value of all weights of a group of NNs. The specific coding method is as follows.

(9) $$\begin{array}{c} \text{particle }\left(i\right)=\left(w_{31}w_{32}w_{41}w_{42}w_{51}w_{52}w_{61}w_{62}w_{63}\right). \end{array}$$

After particle swarm optimization coding, the error criterion function in the BP algorithm is taken as the particle fitness function, and then, the optimization is carried out according to the basic particle swarm optimization process. Finally, the location of the globally optimal particle is the ownership value of the NN. The speed update formula for connecting variables is as follows.

(10) $$\begin{array}{c} v_{ih}⟵w*v_{ih}+c_{1}*\mathrm{rand}*\left(p_{i}-\delta_{ih}\right)+c_{2}*\mathrm{rand}*\left(g-\delta_{ih}\right). \end{array}$$

The output of each node is calculated according to the following equation:

(11) $$\begin{array}{c} Q_{i}^{1}=\mu_{A_{i}}\left(x\right)=\frac{1}{1+{\left[{\left(\left(x-v_{i}\right)/\sigma_{i}\right)}^{2}\right]}^{b}}. \end{array}$$

The two successive changes of weight can be regarded as the change of particle velocity, as shown as follows:

(12) $$\begin{array}{c} Q_{i}^{2}=w_{i}=\mu_{Ai}\left(x\right)\mu_{Bi}\left(y\right),i=1,2. \end{array}$$

The outputs are normalized firing strengths, as shown as follows:

(13) $$\begin{array}{c} Q_{i}^{4}={\bar{w}}_{i}f_{i}={\bar{w}}_{i}\left(p_{i}x+q_{i}y+r_{i}\right),i=1,2. \end{array}$$

The summation of all input signals as the overall output is shown as follows:

(14) $$\begin{array}{c} Q_{i}^{5}=\text{overall output}=\underset{i}{\sum }\;{\bar{w}}_{i}f_{i}=\frac{\sum_{i}\;w_{i}f_{i}}{\sum_{i}\;w_{i}}. \end{array}$$

The inertia weights can be presented as follows:

(15) $$\begin{array}{c} \Delta \omega_{2}=\lambda_{1}e\left(k\right)x_{j}^{\prime }+\lambda_{2}\left[c_{1}r_{1}\left(\omega_{2}\left(b\right)-\omega_{2}\right)+c_{2}r_{2}\left(\omega_{2}\left(g\right)-\omega_{2}\right)\right]. \end{array}$$

However, the current particle swarm optimization algorithm needs a lot of calculation when optimizing the structure of the NN, and it is difficult to meet the requirements for some problems that need online learning. One location is a feasible solution, and the other location is an infeasible solution. When this happens, in order to avoid the problem that the algorithm cannot jump out of the local extreme point due to the loss of important infeasible solution information, in the early stage of evolution, it is allowed to accept the infeasible solution with a certain probability when the function value of the infeasible solution is less than the function value of the feasible solution. However, in the later stage of the algorithm, in order to better carry out local mining, the emergence of the infeasible solution is unbearable; therefore, the probability of accepting an infeasible solution decreases to 0. At this time, it is obviously unreasonable to only consider the size of constraint violation degree and ignore the optimization function of function. Therefore, in this case, how to reasonably balance the relationship between function value and constraint violation degree and select a more reasonable position as the individual optimal guidance position is very important. In order to better evolve continuous variables and discrete variables, this algorithm uses the PSO algorithm with outstanding performance to solve continuous optimization to deal with the optimization of continuous variables, uses the GA algorithm which is mature to solve discrete optimization to deal with the evolution of discrete variables, and organically combines the two by means of collaborative crossover.

## 4. Experiments and Results

Physical exercise refers to the process in which people produce a series of stimuli to various organ systems through scientific activities, promote a series of adaptive changes and reactions to the human body's morphological structure and physiological function, and improve health and physique. Exercise time is usually related to people's exercise load, which is mainly manifested in that if the exercise load is large, the exercise time is short. The analysis of each physical exercise time of college students is shown in Table 1 and Figure 6.

The study found that college students have sufficient physical exercise time. Those who exercise more than 30 minutes each time account for 55% of the total survey, of which 36% are in 30-60 minutes. Boys have more exercise time than girls in general. There are significant differences in physical exercise time between the sexes. Exercise intensity plays a very important role in improving and improving college students' mental health. Different physical exercise intensities will have different effects on the mental health level of college students; that is, the psychological status of students varies with the intensity of physical exercise. The intensity of each physical exercise of college students is shown in Table 2Figure 7 and Figure 8.

The study found that nearly 80% of students said that the intensity of each exercise can reach more than medium intensity, that is, slight sweating all over the body. 36% of the students said they could reach the level of exhaustion every time they exercised. However, studies have shown that the effect of moderate-intensity physical exercise on educating the mental health of college boys is significantly higher than that of low-intensity and high-intensity physical exercise. It is suitable for college girls to use a lower moderate amount of exercise, and the suitability of exercise intensity is the guarantees of good mental health effect. The research shows that the exercise intensity of college boys is generally higher than that of girls, and girls are mainly in the exercise mode below medium intensity. There is a significant difference between exercise intensity and students' gender. Self-stress assessment is to use the self-stress assessment test form to let students fill in the form and answer according to the actual situation, calculate the total score according to the corresponding bisection standard, and then evaluate the degree of stress they feel according to the corresponding score segment. The study found that the mental health level of college students is low, in which only 5% and 25% of the students feel no pressure or feel less pressure, while the number of students with moderate self-pressure accounts for 46% of the total survey, and 18% of the students feel greater self-pressure. The relationship between college students' self-stress test and exercise time is shown in Table 3.

Physical activity is not only beneficial to college students' intellectual growth, but it also has a clear influence on reducing anxiety, building a positive self-concept, and removing psychological barriers, as evidenced by the findings. In the process of exercise, it improves the level of college students' health belief, makes individuals subjectively evaluate psychological stress, and has a great negative impact on health caused by illness so that the health belief that avoiding psychological stress is good for personal health regulates the process of exercise to improve psychological stress. Taking the students in five colleges and universities in Jiangsu Province as the survey object, this paper studies the intervention of physical exercise on college students' mental health by using the methods of literature, investigation, mathematical statistics, and logical analysis.

## 5. Conclusion

College students are a special group, and their physical and mental health is the basis for success. Their physical appearance and health are directly tied to the future health, scientific, and technical benefits of high-tech teams. We require physical exercise to strengthen our bodies because our daily studies and lives prevent us from moving for long periods of time. This research suggests a physical exercise intervention based on enhanced NN that has an effect on college students' mental health. To sum up, the appropriate sports plan can help college students carry out scientific and reasonable exercises. This kind of physical exercise mode has stronger pertinence and is effective in improving and improving the mental health level of college students.

At present, medical psychology has achieved certain results in the diagnosis and treatment of mental diseases, but the particularity of physical exercise cannot be compared with other ways to improve and treat mental diseases. For college students, it is more effective and useful. College students are frequently impacted by emotional oscillations and excessive mental tension due to the quick speed of work and living in today's culture, as well as severe rivalry. College students can formulate appropriate physical exercise methods to improve their mental health level according to their own physical conditions, health status, interests, and hobbies and make timely adjustments and interventions for their psychological and emotional adverse reactions, so as to make their physical and mental relaxation moderate and always maintain a relatively stable state. Because physical exercise has high application value and theoretical research value to promote the level of mental health, we should constantly explore this field and study more effective means and methods to improve the level of mental health.

## Figures and Tables

**Figure 1:** The relationship between physical exercise and students' mental health.

**Figure 2:** The mechanism of physical exercise affecting psychological stress.

**Figure 3:** The impact of an exercise intervention on college students' health beliefs.

**Figure 4:** The basic flow of particle swarm optimization algorithm.

**Figure 5:** Particle swarm optimization NN structure diagram.

**Figure 6:** Analysis of physical exercise time of college students.

**Figure 7:** The intensity of each physical exercise of college students.

**Figure 8:** The relationship between college students' self-stress test and exercise time.

**Table 1:** Analysis of physical exercise time of college students.

Exercise time	Man	Woman	Total
10 min~ 30 min	17%	28%	45%
30 min~ 60 min	21%	15%	36%
More than 60 minutes	13%	6%	19%
Total	51%	49%	100%

**Table 2:** The intensity of each physical exercise of college students.

Exercise time	Man	Woman	Total
High strength	21%	15%	36%
Medium strength	23%	20%	43%
Small strength	6%	9%	15%
Other	1%	5%	6%
Total	51%	49%	100%

**Table 3:** The relationship between college students' self-stress test and exercise time.

Exercise time	High pressure	Medium pressure	Low pressure
10 min~ 30 min	55	64	42
30 min~ 60 min	32	57	66
More than 60 minutes	20	33	76

## Data Availability

The datasets used during the current study are available from the corresponding author on reasonable request.
